# Application of a Fast RCNN Based on Upper and Lower Layers in Face Recognition

**DOI:** 10.1155/2021/9945934

**Published:** 2021-09-24

**Authors:** Lin Jiang, Jia Chen, Hiroyoshi Todo, Zheng Tang, Sicheng Liu, Yang Li

**Affiliations:** ^1^Ministry of Science and Education, Toyama University, Toyama 930-8555, Japan; ^2^Shandong Key Laboratory of Language Resources Development and Application, Ludong University, Yantai 264025, China; ^3^Wicresoft Japan, Tokyo 190-0155, Japan; ^4^School of Mechanical and Electrical Engineering and Automation, Shanghai University, Shanghai 200444, China

## Abstract

With the development of society, deep learning has been widely used in object detection, face recognition, speech recognition, and other fields. Among them, object detection is a popular direction in computer vision and digital image processing, and face detection is a focus of this hot direction. Although face detection technology has gone through a long research stage, it is still considered as one of the more difficult subjects in human feature detection technology. In addition, the face detection technology itself has two sides, imperceptibility and complexity of the environment, and other defects cause the existing technology to be unable to accurately recognize faces of different proportions, obscured and different postures. Therefore, this paper adopts an advanced deep learning method based on machine vision to detect human faces automatically. In order to accurately detect a variety of human faces, a multiscale fast RCNN method based on upper and lower layers (UPL-RCNN) is proposed. The network is composed of spatial affine transformation components and feature region components (ROI). This method plays a vital role in face detection. First of all, multiscale information can be grouped in detection, so as to deal with small areas of the face. Then, the method can use the inspiration of the human visual system to perform contextual reasoning and spatial transformation, including zooming, cutting, and rotating. Through comparative experiments, the analysis results show that this method can not only accurately detect human faces but also has better performance than fast RCNN. Compared with some advanced methods, this method has the advantages of high accuracy, less time consumption, and no correlation mark.

## 1. Introduction

At present, face detection technology has been widely used in many fields such as security, campus, and finance [1]. With the progress of society and the further maturity of technology, face detection technology will inevitably be applied to more fields [2]. However, the human face is a very common but very complex pattern, which contains a lot of information [3]. It is a difficult problem to distinguish human faces from other objects in a complex background image, and due to changes in the proportions, poses, facial expressions, lighting, image quality, age, and occlusion of the face, face detection becomes more difficult, as shown in Figure 1. Therefore, in order to complete the robustness of the detection method, the designed detection algorithm must consider the possible interference caused by various complex backgrounds of the face [4].

Faster R-CNN is a method based on the fast regional convolutional network. It can effectively improve the detection efficiency and accuracy by using the deep convolutional network to effectively extract and classify the object to be detected [5]. Compared with traditional face detection technology, Faster R-CNN adopts the technology of region of interest pooling (ROI pooling), so that the network can share the calculation results, thereby speeding up the model [6]. The traditional CNN structure can maintain a certain degree of translation and rotation invariance for a specific location in the input image. This kind of spatial invariance is only in the local area of the input image, and the entire image cannot achieve the invariance of the overall spatial rotation in the stacked local area [7]. Because the pooling layer in the CNN structure has many limiting factors, for example, much useful information will be lost when extracting features, and the input data are only a partial operation [8]. The feature map in the middle of the CNN framework will produce large distortions; as a result, it is difficult for CNN to implement spatial transformations such as image rotation and scaling [9]. The feature map generated in the process of CNN's feature extraction is not an overall transformation of the input data, which is more restrictive [10]. At the same time, when the amount of data in the training face data set is huge, a large number of candidate regions will be generated and occupy the space of the disk. And when the candidate regions are transmitted to the CNN, they will be normalized in advance to cause the loss of information [11]. Each candidate region is placed in the network, causing the same feature to be repeatedly extracted and wasting resources [12].

The spatial affine transformation module is a dynamic mechanism that can actively perform a spatial transformation on the input image and perform an overall transformation on the entire image, including transformations such as scaling, cropping, and rotation. The affine transformation module is mainly divided into three parts: positioning network, grid generator, and sampler. This module can effectively solve the impact of changes in scale and viewing angle on the accuracy of face recognition.

The network in this paper is an improvement on the traditional Faster R-CNN, and a multiscale fast RCNN method based on the upper and lower layers is proposed, which can detect small targets robustly in different scales, poses, and environments [13]. The experimental results show that the multiscale fast RCNN based on the upper and lower layers has better detection performance than the fast RCNN while maintaining the same test cost. Compared with the most advanced face detection methods at present, the improved method in this paper can accurately detect faces in different poses in various environments.

The contributions and originality of this paper are summarized as follows: (1) For the first time, a new space radiological transformation is proposed to improve the detection ability of the original Faster-RCNN. The spatial affine transformation recognizes the face parts by detecting meaningful areas in the image, thereby improving the detection effect of the original network on small parts of the face. The experimental results also verify that UPL-RCNN's face detection is improved compared to other networks. (2) A method of combining upper and lower layers is proposed. The upper layer adopts the affine transformation strategy, and the lower layer adopts the characteristic region strategy. It enables the original network to robustly detect small targets in different scales, different poses, and different environments. (3) The affine space transformation uses feature fusion, which strengthens the continuity of actions and can better improve the ability of face recognition.

## 2. Related Work

Face detection is a hot topic in the field of computer vision [14]. With the increasing demand, face detection technology has received widespread attention from universities, scientific research institutes, and enterprises, and many new face detection methods have emerged. It can be used as a pre-work in many fields such as face recognition and face tracking [15]. Therefore, how to improve the effect of face detection under existing conditions has become a common research goal of many institutions. In addition, the quality of face images and the level of data set production also have a great influence on face detection [16]. In recent years, many excellent models have appeared in the field of face detection. The earliest excellent model capable of real-time detection is Viola-Jones [17]. This framework uses rectangular Haarlike features in the cascaded AdaBoost classifier for the first time, thus realizing real-time face detection. However, it has some disadvantages, such as the relatively large feature size, and the effect of dealing with nonfrontal faces and faces in complex environments is not very good [18]. In order to solve the defect of the VJ algorithm, improvements have been made in the use of features, such as HOG, SIFT, SURF, and ACF. There are also changes in the classifier [19]. For example, Dlib C++ Library uses SVM as the classifier, and some methods use random forest as the classifier [5].

Then came the Deformable Parts Model (DPM). This model is based on the improvement of the HOG descriptor, mainly to solve the problem of inaccurate detection caused by different angles of the object [4]. DPM has achieved good detection results in many detection fields and has become the best detection model. It has also been the best model in the field of face detection until the emergence of the CNN model.

In recent years, with the continuous development of deep learning models, the combination of excellent face detection models and deep learning models has made face detection better [20]. For example, Yunzhu Li used an end-to-end multitask learning framework that integrates ConvNet and 3D mean face model in his paper and achieved good results. Recently, due to the rise of the Faster-RCNN model, many face detection models have begun to be combined with the Faster-RCNN model. For example, Hongwei Qin used this model in his paper, and the experiment used the FDDB data set and achieved good results. More models are improvements to the Faster-RCNN model to make their models more suitable for face detection in complex backgrounds. For example, the model designed by Wan et al. in conjunction with ResNet and OHEM (Online Hard Example Mining) has achieved excellent results on many face data sets. Li et al. designed a real-time visual tracking model based on convolutional neural networks, which can track target objects in real time [21]. Garcia-Ortiz et al. proposed a system to realize the detection and segmentation of human contours [22]. Sun et al. proposed a face detection scheme using deep learning [23]. Moreover, Xudong Sun used strategies of the Feature Concatenation, Hard Negative Mining, and Multiscale Training to improve the model on the basis of Faster R-CNN and has achieved good results on the FDDB data set [24].

There are also many people who use human visual mechanisms to design models. For example, the most famous is salient object detection, which uses human attention mechanism to design models. The main idea is to use the biological model proposed by Koch and Ullman to integrate features with several other models to explain the human visual search strategy [25]. The visual input is first divided into a series of feature topographic maps, and then in each map, different spatial positions obtain saliency through competition, and only the positions that stand out from the surroundings can be retained. All feature maps are input to the advanced saliency map in pure BU mode, which encodes the local conspicuousness of the entire visual scene [26]. In primates, it is believed that this picture exists in the posterior parietal cortex and also in the pulvinar nuclei of thalamus [27]. The saliency map of the model is considered to be the internal motivation that produces attention shift. Therefore, this model shows that the saliency of BU can guide attention shift, without TD. This model can be processed in parallel to increase the speed of calculation and can add weights to features according to their importance. The more important the features, the greater the weight [28]. Xiaoning Zhang's paper proposes a new attention-guided network model that selectively integrates multilevel contextual information in an incremental manner. In addition to simulating the human attention mechanism, there is some research work that analyzes the importance of the information around the face object in judging the position of the face [29–33].

This article is based on the Faster R-CNN model, and the CNN part of the Faster R-CNN model uses ResNet50 as the feature extractor. This is because the residual network has the best comprehensive performance in feature extraction, and the two most important points in the design model are the environment around the face and the introduction of human attention mechanism. The surrounding environment of the human face considers the human face, because in a complex background, there will be a lot of occlusion, such as lighting or resolution issues. Therefore, considering the influence of these factors on face detection, this paper uses spatial affine transformation to improve the Faster-RCNN network model. By detecting meaningful areas in the image, the human body's movements are identified by parts, so as to improve the accuracy and detection speed of the original model.

## 3. The Proposed Method

The performance of Faster R-CNN on the PASCAL VOC data set has reached the world's leading level and can detect human, animal, vehicle, and other targets. These targets usually occupy a large area in a picture. But the goal of this article is to perform face detection under different backgrounds and different forms of challenging conditions, such as small faces, occluded faces, faces with different expressions, faces with different poses, and faces with different proportions. In this case, when the existing Faster R-CNN model performs face detection, the feature map obtained by its RoI layer has only one scale, which leads to a high rate of missed detection of face detection. In addition, overfitting is more likely to occur when training in broader data sets and real data sets, resulting in low accuracy of detection. The method proposed in this paper can effectively solve this problem.

### 3.1. Faster R-CNN Model

Faster R-CNN is the best method for object detection among all the improved algorithms based on R-CNN. It searches for candidate areas by introducing a region proposal network (RPN) instead of selective search. The feature maps obtained from the input pictures are passed through the convolutional neural network and then these maps are sent to the regional suggestion network. The regional proposal network filters out the anchor points with the highest classification confidence from a large number of preset anchor points, determines these anchor points as candidate frames, and then sends them to the RoI pooling layer together with the feature map to obtain the pooled region of interest features. Finally, these pooled features are sent to the fully connected layer and then classification and border regression are performed.

An important concept in the regional proposal network is the anchor point. As the name suggests, the anchor point is the point where the anchor position is located. It is composed of a series of preset borders of different sizes. As shown in Figure 2, the RPN network can be seen as a feature map. By sliding the window on the feature map through the frame, a series of anchor points are generated. For example, the red box indicates the position of the current candidate area on the feature map. The location of this area is mapped to the size and shape of the corresponding area on the original image. K anchor points of different sizes are set. Then from left to right and top to bottom on the feature map, each point corresponds to generating K anchor points, until the complete feature map is traversed. Then, for all these anchor points, a classifier will be used to give a confidence in the foreground, the position of the anchor will be corrected by regression, and finally the 2000 anchor points with the highest confidence will be selected as the candidate frame, together with the feature map send it to the RoI pooling layer.

### 3.2. New Spatial Affine Transformation

By calculating the gradient along the contour of the human face, the nontarget face and the target face can be distinguished well according to the shape. Let *X* be a candidate rectangular region and set the position of the pixel on the side of the rectangle as (*x*_*i*_, *y*_*i*_). For the plane change of the face during tracking, affine transformation is used to describe the change of its contour. The shape space of the initial rectangle contour change can be described by the shape parameter vector *S*; then,

(1) $$\begin{array}{c} \left[\begin{array}{c} x_{i}^{\prime }\\ y_{i}^{\prime } \end{array}\right]=\text{WS}+\left[\begin{array}{c} x_{i}\\ y_{i} \end{array}\right]. \end{array}$$

Among them, $\left[\begin{array}{c} x_{i}\\ y_{i} \end{array}\right]$ is the starting rectangular area, and *W* is the shape matrix.

As the dimension of the rectangular space is 2*N*, if the dimension of the introduced shape space is *N*_*s*_, then *S* is the matrix of *N*_*s*_ × 1, and *W* is the matrix of 2*N* × *N*_*s*_. Affine transformation is usually represented by 6 degrees of freedom, so *N*_*s*_=6. The shape matrix *W* is defined as

(2) $$\begin{array}{c} W=\left[\begin{array}{ccc} 1 & 0 & x_{i}\\ 0 & 1 & 0 \end{array}\;\begin{array}{ccc} 0 & 0 & y_{i}\\ y_{i} & x_{i} & 0 \end{array}\right]. \end{array}$$

Through the shape model of the target, the parameter vector *S* of the target can be obtained, and *S* can be expressed by the following formula:

(3) $$\begin{array}{c} \;S=\left(O_{x}^{\prime },O_{y}^{\prime },I_{x}^{\prime }\cos\;\theta^{\prime }-1,\;I_{y}^{\prime }\cos\;\theta^{\prime }-1,\;-I_{y}\sin\;\theta^{\prime },-I_{x}\sin\;\theta^{\prime }\right).\; \end{array}$$

Here, *O*_*x*_′ and  *O*_*y*_′ is the change of the target center point; *θ* is the angle of the target contour change; and *I*_*x*_′ and  *I*_*y*_′ are the proportional changes of the target in the *x* and *y* directions, respectively.

Each face has its own posture. For each face, it can be set to *N*, and *O* is used to represent the different postures of each face. The shape parameter *I*^*i*^ can be calculated by the posture. The position (*x*_*i*_′,  *y*_*i*_′) of each point of the rectangular contour is calculated by the shape parameter *O* after affine transformation. Sample *N* points (*x*_1_^*i*^,  *y*_1_^*i*^, *i*=1,…, *N*), on the contour, draw a normal at each point, and calculate the gradient value *M*_*j*_(*j*=1,2,…, *N*) of each normal. Comparing the distance between the pixel point and the pixel point of the maximum gradient (*x*_2_^*i*^,  *y*_2_^*i*^,  *i*=1,…, *N*), the similarity between the required contour and the real contour can be calculated. This paper proposes a new method of measuring the distance between each other, using the distance between each other to express the similarity. When the environment is known, the relative distance between two points *x*_*i*_ and *x*_*j*_ is defined as follows:

(4) $$\begin{array}{c} d_{\text{kmnrd}}\left(x_{i},x_{j};k,\mu_{i},\mu_{j}\right)=\mu_{i}\times \text{NNR}\left(x_{i},x_{j};k\right)+\mu_{j}\times \text{NNR}\left(x_{j},x_{i};k\right). \end{array}$$

Among them,

(5) $$\begin{array}{c} \text{NNR}\left(x_{i},x_{j};k\right)=\frac{d^{\prime }\left(x_{i},x_{j}\right)}{\text{BD}\left(x_{i};k\right)}, \end{array}$$

(6) $$\begin{array}{c} \text{BD}\left(x_{i};k\right)=\frac{1}{k}\overset{k}{\underset{j=1}{\sum }}d^{\prime }\left(x_{i},x_{j}\right). \end{array}$$

Here, *d*′(*x*_*i*_, *x*_*j*_) represents a certain distance commonly used between *x*_*i*_ and *x*_*j*_, such as the commonly used Euclidean distance. BD(*x*_*i*_; *k*) is the k-nearest neighbor base distance of *x*_*i*_ and represents the distance reference of *x*_*i*_. NNR(*x*_*i*_, *x*_*j*_; *k*) represents the ratio of the distance between the points *x*_*i*_ and *x*_*j*_ relative to the distance of the *k*-nearest neighbor base of *x*_*i*_, and the calculation of the ratio is effective to offset the influence of the unit of measurement. *μ*_*i*_ and *μ*_*j*_, respectively, represent weights, which are suitable for situations where the importance of data is different. In the detection task, due to the limited knowledge of the data, it is generally considered that the importance of the data in the initial trial is the same, so it is only necessary to set the same value. According to the definition formula, the symmetry is satisfied when *μ*_*i*_=*μ*_*j*_=*μ*:

(7) $$\begin{array}{c} d_{\text{kmnrd}}\left(x_{i},x_{j};k,\mu ,\mu \right)=\mu \times \left(\text{NNR}\left(x_{i},x_{j}\right)+\times \text{NNR}\left(x_{j},x_{i}\right)\right)=d_{\text{kmnrd}}\left(x_{j},x_{i};k,\mu ,\mu \right). \end{array}$$

Compared with the original MND, it no longer only uses the nearest neighbor ranking position between the data points, but more uses the distance between the data points. At the same time, starting from *k*-nearest neighbors, more global information of data points is used. The *k*-nearest neighbor base distance of *x*_*i*_ represents the distance measurement standard of each point.

Then, the observed probability density function can be expressed as Compared with the original MND, it no longer only uses the nearest neighbor ranking position between the data points, but more uses the distance between the data points. At the same time, starting from *k-*nearest neighbors, more global information of data points is used; The *k*-nearest neighbor base distance of *x*_*i*_ represents the distance measurement standard of each point.

Then, the observed probability density function can be expressed as

(8) $$\begin{array}{c} P\left(z_{k}\;|\;x_{k}^{i}\right)\exp\left\{-\frac{1}{2\sigma^{2}}d\right\}. \end{array}$$

After determining its color model, the observation probability density function is

(9) $$\begin{array}{c} P\left(z_{k}\;|\;x_{k}^{i}\right)=\frac{1}{\sqrt{2\pi }}\exp\left\{-\frac{d^{2}\left(p\left(x\right),q\right)}{2\sigma^{2}}\right\}. \end{array}$$

There are various fusion methods for multicharacter information, and the democratic fusion strategy is adopted here. If a certain information is reliable in the current frame, its weight will be large. This method increases the complementarity between information and improves the robustness of the observation target. The weighted combination of color model and shape model information can be expressed as

(10) $$\begin{array}{c} P\left(z\;|\;x\right)=\omega^{c}p\left(z^{c}|x\right)+\omega^{g}p\left(z^{g}|x\right). \end{array}$$

Among them, *ω*^*c*^ and *ω*^*g*^, respectively, represent the weighting of color information and shape information and represent the reliability of the information.

Finally, this article uses maximum likelihood estimation to represent the state of the target, and the formula is as follows:

(11) $$\begin{array}{c} \hat{X}=\begin{array}{c} \arg\max\\ x \end{array}\left\{p\left(z|x\right)\right\}. \end{array}$$

### 3.3. Multiple-Scale Faster-RCNN Based on Upper and Lower Layers

Due to differences in occlusion, proportions, posture, and lighting brightness of human faces, in this case, the existing Faster-RCNN mainly has two problems: (1) small faces in photos that cannot be detected. (2) For different poses and different backgrounds, the accuracy of face detection is low. Therefore, this paper uses a new affine space to propose a multiscale fast RCNN method based on upper and lower layers. The new affine space is spatially operated on the data in the Faster-RCNN framework. After modification, it can be simply inserted into the existing network, and the integrated structure can still be trained end-to-end without additional supervision or back-propagation for tuning training. The network structure diagram is shown in Figure 3.

In different situations, the size, position, and shape of the face may be very different, which belongs to the intraclass and interclass differences in face recognition. And there will be some objects in the image that are similar to human faces but have nothing to do with face detection, which can be ignored. The new spatial affine transformation can automatically obtain the region of interest. Therefore, a new spatial affine transformation is added to the convolutional layer of the Faster-RCNN structure to detect the face by region. Through experimental tests, six new spatial affine structures have the best effect on face recognition. As shown in Figure 4, the network structure of this paper first performs spatial affine transformation on the input face to correct the spatial position of the face. Six spatial affine transformation structures are used to extract features of the face after the convolutional layer, combine multiple regional features for face detection, and then use the alternate structure of the convolutional layer and the pooling layer to extract more advanced facial features.

After building the Faster-RCNN framework and image input, the extracted features are fused. Feature fusion is introduced to enhance the detection of human faces, so that the model can obtain better performance. This article uses the following method for fusion. Assume that *Y* is used to represent the final feature of the input image, then the formula of *Y* is

(12) $$\begin{array}{c} Y=\omega_{1}X_{1}+\omega_{2}X_{2}. \end{array}$$

Here, *X*_1_ represents the spatial feature, *X*_2_ represents the attribute feature, and *ω*_1_ and *ω*_2_, respectively, represent the weight of the two features and the sum is 1. The above formula can calculate the weighted sum of spatial features and attribute features. The output after feature fusion is used as the input of the softmax layer for face recognition.

### 3.4. Model Training

The parameter settings of the UPL-RCNN network model will directly affect the detection accuracy and detection speed of the model. If the design of the front-end network model is too complicated, it will lead to a lower recall rate and also affect the face detection speed; if the back-end network model is designed too simple, it will lead to a decline in detection accuracy. Therefore, in the UPL-RCNN model, the setting of network parameters is very important. In order to obtain better parameters when training the network model, this paper uses multiple iterations and ten-fold cross-validation methods to train the UPL-RCNN model, which can effectively avoid overfitting problems while ensuring the detection rate and detection speed.

In the training process, the UPL-RCNN model is trained using the WIDER FACE data set. In order to avoid the overfitting problem of the UPL-RCNN model and improve the reliability and stability of the model, this paper uses the ten-fold cross-validation method in cross-validation method to train the model. Using ten-fold cross-validation, first, divide the training positive sample and negative sample data sets into 10 equally and use 9 of them to train the UPL-RCNN model in turn, use the remaining 1 as the test data set to test the model, and finally the average of the results of 9 training and 1 test is used as an estimate of the effectiveness of the UPL-RCNN model, and the cross-validation is repeated 10 times to ensure that each subsample is verified once, thereby improving the detection accuracy of the network model. At the same time, the UPL-RCNN model parameters are repeatedly adjusted by using multiple iterations. When the number of iterations reaches 1,000, the model converges. Therefore, the number of iterations for the network model during training is 1, 100, 500, and 1,000. The method of this paper is compared with other advanced models in terms of both experimental error and training time. The comparison of the error and training time under different iteration times is shown in Table 1. With the increase of the iteration times and the adjustment of the parameters, the error gradually decreases. The specific parameter settings are shown in Table 2.

## 4. Experimental Results

In order to verify the results of the multiscale fast RCNN method based on the upper and lower layers on the face style, this paper uses the WIDER FACE data set and real-life shooting data for experiments. The comparison algorithms include Faster-RCNN, Two-stage CNN, Single Shot Detector, R-FCN, Hyper Face, and Aggregate Channel Features (ACF). In this article, the multiscale fast RCNN method based on the upper and lower layers is implemented in python. All algorithm experiment environments are Win10 64 bit operating system, python software, 16G memory, Intel (R) Xeon (R) CPU E3-1231 v3@3.40GHz. The following Section 4.1 briefly describes the experimental data set information and evaluation criteria, Section 4.2 gives the face detection results and corresponding analysis on the WIDER FACE data set, and Section 4.3 gives the face detection results and corresponding analysis on the subway station data set.

### 4.1. Description of the Data Set

Because the WIDER FACE data set is too large, we randomly selected 40%, 10%, and 50% on the WIDER FACE data set as the training set, validation set, and test set for training and testing. This data set contains 32,203 images, with a total of 393,703 face tags. Different expressions, illumination, invalid, occlusion, and pose of each face are marked. This division is very beneficial for training and testing. The detection part of the test data set is shown in Figure 5.

After completing the modeling, we need to evaluate the effect of the model. The evaluation indicators that are often used are Accuracy, Recall, F-Measure, etc., and this article uses Accuracy and Recall:

(a) Accuracy refers to the percentage of correct prediction results in the total sample, which depends on TP (true positive) and FP (false positive). TP refers to predicting a positive class as a positive class number. FP refers to predicting a negative class as a positive class number false positive, that is,
  (13) $$\begin{array}{c} P=\frac{\text{TP}}{\text{TP}+\text{FP}}. \end{array}$$
(b) Recall is only for the original sample, and its meaning is the probability of being predicted as a positive sample in the actual positive sample, which depends on TP and FN (false negative). FN refers to the number of samples that predict the positive class as the negative class.
  (14) $$\begin{array}{c} R=\frac{\text{TP}}{\text{TP}+\text{FN}}. \end{array}$$
(c) PR is an index to measure the accuracy of the algorithm in Object Detection algorithm, which involves two concepts: Precision of Precision and Recall. For object detection task, Precision and Recall can be calculated for each object. After multiple calculations/tests, a P-R curve can be obtained for each class, and the area under the curve is the value of AP. This means that the AP of each class can be averaged to get the value of PR. The size of PR must be in the interval [0, 1].

(15) $$\begin{array}{c} \text{AP}=\int_{0}^{1}P\left(R\right)\text{d}R=\overset{n}{\underset{k=0}{\sum }}P\left(k\right)\Delta R\left(k\right), \end{array}$$

(16) $$\begin{array}{c} \text{PR}=\frac{\sum_{i=1}^{c}{\text{AP}}_{i}}{C}. \end{array}$$

In the object detection experiment, we hope that the ideal condition of the test results is high accuracy and high recall. However, in actual experiments, accuracy and recall are often in conflict in some cases. In some extreme cases, for example, when only one result is returned, the accuracy rate is 100%, but the recall rate is very low. When returning all the results, the recall rate is 100%, but the accuracy rate will be very low. Therefore, we cannot just look at the correct rate or the recall rate. We should determine whether accuracy or recall is more important based on the actual situation. Therefore, in order to avoid a single test standard from affecting the results of data analysis, it is necessary to use an Accuracy-Recall curve for analysis.

### 4.2. Experimental Results and Analysis of the WIDER FACE Data Set

This article compares experiments with Faster-RCNN, Two-stage CNN, Single Shot Detector, R-FCN, Hyper Face, and Aggregate Channel Features (ACF) models to prove the effectiveness of this model. All models use the same training set and test set. The training difficulty is set to three levels, which are easy, medium, and difficult.  Figure 6 shows the PR curves of the model in this paper and the comparison model. This figure compares the performance of the above face detection methods very intuitively.

It can be seen from Figure 4 that the UPL-RCNN model has the highest accuracy rate compared to other models. For the UPL-RCNN model, its performance is significantly better than Faster-RCNN, indicating that the multiscale fast RCNN method based on the upper and lower layers can better detect faces. Compared with two-stage, because of its detection characteristics, the selection range of the input image size is relatively loose. For the two-stage operation of serial candidate frame selection and target positioning and classification, the accuracy of the model in this paper is greatly improved. The model in this paper can input larger scale images compared to the Single Shot Detector model, and because this method uses multiscale feature fusion operation for detection, the detection accuracy has been greatly improved. However, there are corresponding shortcomings, the network structure is more complicated, and the detection time has a certain increase. Compared with the R-FCN model, because it uses a multiscale IOU to filter the suggestion frame, it adds a detector to the entire network framework compared to the model in this paper, so the method in this paper has improved the accuracy of detecting faces. Compared with the Hyper Face model and the ACF model, the UPL-RCNN model can further integrate various features through the residual module, so the accuracy is relatively high. The UPL-RCNN model can mainly recognize small faces, occluded faces, and faces in different backgrounds, so it can be improved in accuracy compared to other models.

This paper selects the data in the WIDER FACE data to form a new data set of easy, medium, and hard and then conducts test experiments, respectively, to further prove the overall performance of the UPL-RCNN model. Finally, the baseline method of each model was used for evaluation, and the results are shown in Table 3. Because there are a large amount of small target face data in the hard subset of the WIDER FACE data set, it is fully proved that the method in this paper is superior to other methods in the detection of various types of faces such as small faces. It also has very good robustness on the easy and medium subsets.

### 4.3. Analysis of Face Detection Results in the Subway Station Data set

In order to fully prove the effectiveness of the multiscale fast RCNN method based on the upper and lower layers on the face detection results, we apply the model in this paper to the face detection in real scenes such as subway stations. In the process of detecting human faces in subway station passenger flow, especially in the morning and evening peak hours, when the passenger flow density is high, the situation of mutual occlusion of faces between passengers is more serious. Therefore, we select 5000 images obtained through data enhancement and divide them into easy, medium, and hard data sets and continue to fine-tune the training on the model.  Figure 7 shows the face detection results.  Figure 8 shows the PR curves of this model and other models.

From the comparison curve, it can be seen that the UPL-RCNN model is more effective in face detection in real data sets than Faster-RCNN, Two-stage CNN, Single Shot Detector, R-FCN, Hyper Face, and Aggregate Channel Features (ACF). Among them, the UPL-RCNN model has an increase of 16.2% compared with the Faster-RCNN model, and the Faster-RCNN model is much higher than other models in face detection. Therefore, the model in this paper is effective in detecting small faces and covering faces.

## 5. Conclusion

The Faster-RCNN model has the problem of low face detection rate under complex background, different scales, and different poses. Aiming at such problems, this paper proposes an improved model UPL-RCNN model. The model is composed of spatial affine transformation components and characteristic region components and grouping multiscale information to process small regions of human faces. Then use the inspiration of the human visual system to carry out contextual reasoning and spatial transformation. From the experimental results of the WIDER FACE data set and the subway station data set, it can be seen that this paper has a higher advantage than other models in recognizing faces of different proportions and different poses, but it has not yet reached the optimal time consumption. Therefore, how to improve the time consumption of the model under a huge data set is a work that needs further research.

## Figures and Tables

**Figure 1:** WIDER FACE data set categories.

**Figure 2:** RPN network structure diagram.

**Figure 3:** Network structure diagram.

**Figure 4:** Affine structure.

**Figure 5:** WIDER FACE data set analysis.

**Figure 6:** WIDER FACE data set PR curve comparison results.

**Figure 7:** Face detection results.

**Figure 8:** Comparison results of PR curves of subway station data sets.

**Table 1:** Error and time comparison under different iteration times.

model	1 time		100 times		500 times		1000 times	
	Error/%	Time/s	Error/%	Time/s	Error/%	Time/s	Error/%	Time/s
Hyperface	48.27	97	4.87	198	0.93	869	0.86	2008
Aggregate channel features	35.42	86	4.19	150	0.81	812	0.79	1643
R-FCN	33.29	77	3.65	109	0.71	648	0.61	1200
Single shot detector	30.15	75	3.24	100	0.66	620	0.52	1105
Two-stage CNN	30.58	63	2.93	97	0.59	582	0.38	974
Faster-RCNN	27.34	51	2.42	84	0.47	409	0.21	811
UPL-RCNN	23.62	42	2.21	76	0.31	378	0.09	723

**Table 2:** Initial settings of specific parameters of the pretraining model.

Pretrained model	Parameter	Fine-tuning
UPL-RNN	Num_classes	36
	Batch_size	1
	Initial_learning_rate	0.0003
	Momentum_optimizer_value	0.9
	Num_steps	1000

**Table 3:** Comparison of per class AP.

	Gymn	Boat	Ball	Tenn	Socc	Grou	Inte
HyperFace	70.8	50.8	61.9	69.3	69.9	71.4	59.5
Aggregate channel features	74.9	55.9	63.7	72.5	70.6	70.7	62.8
R-FCN	72.4	57.3	65.3	71.2	74.1	69.8	61.1
Single shot detector	70.5	53.4	64.2	70.1	71.2	68.3	60.0
Two-stage CNN	75.0	60.2	64.7	66.7	72.7	70.6	61.8
Faster-RCNN	75.6	57.4	68.3	74.4	74.5	72.5	68.0
UPL-RCNN	76.8	63.0	70.1	75.9	76.8	77.9	69.7

## Data Availability

The data used to support this study are available in the following link: https://shuoyang1213.me/WIDERFACE/.
